RETRACTED

# Pathological Roles of Interleukin-22 in the Development of Recurrent Hepatitis C after Liver Transplantation

**DOI:** 10.1371/journal.pone.0154419

**Published:** 2016-04-28

**Authors:** Yinjie Gao, Hui Ren, Fanping Meng, Jin Li, Eddie Cheung, Hanwei Li, Jingmin Zhao, Hongling Liu, Zhenwen Liu, Min Zhang

**Affiliations:** 1 Liver Transplantation and Research Center, 302 Military Hospital, Beijing, China; 2 Department of Infectious Diseases, Medical School of Chinese PLA, Beijing, China; 3 Liver Cirrhosis and Research Center, 302 Military Hospital, Beijing, China; 4 California Pacific Medical Center, San Francisco, California, United States of America; 5 University of California at Davis school of medicine, Sacramento, California, United States of America; 6 Department of Pathology and Hepatology, 302 Military Hospital, Beijing, China; SAINT LOUIS UNIVERSITY, UNITED STATES

## Abstract

**Objective:**

The aim of this study was to longitudinally evaluate and analyze the role of interleukin-22-producing CD4 positive cells (IL-22) in the pathogenesis of Hepatitis C Virus recurrence after Orthotopic Liver Transplantation (HCV-OLT).

**Methods:**

15 HCV-OLT, 15 age- and gender- matched non-HCV post-OLT (OLT) and 15 hepatitis C virus infected (HCV) patients were enrolled into our study from the liver transplantation and research center at Beijing 302 Hospital. We determined the frequencies of IL-22 using flow cytometry and expression of IL-22 mRNA using PCR in peripheral blood and liver tissue. We also divided HCV-OLT patients into rapid fibrosis progression (RFP) and slow fibrosis progression (SFP), examined IL-22 cells and analyzed the correlations between IL-22 frequencies and liver injury, fibrosis and clinical parameters. Moreover, we investigated the role of IL-22 in Human Hepatic Stellate Cells (HSCs).

**Results:**

The levels of serum IL-22, frequencies of IL-22 producing cells in peripheral blood mononuclear cells, and expression of IL-22 mRNA and protein in the liver in the HCV-OLT group were significantly higher than that in the HCV and OLT groups. Furthermore, eight (53.3%) patients developed RFP after two years; another three patients were diagnosed liver cirrhosis. The frequencies of IL-22 were much higher in RFP compared with SFP, while no significant difference existed between OLT and SFP. Intrahepatic IL-22 positive cells were located in fibrotic areas and significantly correlated with α-smooth muscle actin (α-SMA) and fibrosis staging scores, not with grading scores and HCRVNA. *In vitro*, IL-22 administration prevented HSCs apoptosis, promoted HSCs proliferation and activation, up-regulated the expression of HSC-sourced growth factors including α-SMA, TGF-β and TIMP-1, and increased the production of liver fibrosis markers including laminin, hyaluronic acid and collagen type IV.

RETRACTED

**Conclusion:**

Peripheral and intrahepatic IL-22 is up-regulated and plays a pathological role in exacerbating liver fibrosis by activating HSCs in HCV-OLT patients, which may predict RFP and serve as an attractive target for anti-fibrotic therapy.

## Introduction

Chronic hepatitis C virus (HCV) infection is a major public health problem, with an estimated 130 to 170 million people currently infected worldwide and an additional 3 to 4 million are newly infected each year [1]. The increasing burden of this epidemic is reflected by increasing prevalence of end-stage liver disease (ESLD) [2] and hepatocellular carcinoma (HCC) [3]. HCV-related disease represents the most common indication for orthotopic liver transplantation (OLT) [4], accounting for around 40% of all cases on the United States waiting list [5]. Furthermore, projections have showed a constant increase in the number of patients with HCV-related ESLD who will be listed for OLT over the next 10 years [6]. Unfortunately, almost all patients become HCV recurrence after OLT (HCV-OLT) and graft reinfection is universal after liver transplantation [7], which leads to accelerate graft loss and diminish patient survival with liver cirrhosis (LC) within five years of post-transplantation in approximately 20% and within ten years in 50% [8], compared with less than 5% of non-transplantation HCV patients. In a recent review of the Organ Procurement Transplant Network/United Network of Organ sharing (OPTN/UNOS), three-year survival was at 78% for 7,459 anti-HCV positive patients [9]. Several certain pre-OLT factors such as donor age, severity of illness, as well as recipient and donor race have been associated with an increased risk of disease progression and worse post-OLT outcomes [10–20]. After OLT, persistent low-level inflammation and loss of viral control mechanisms from systemic immunosuppression are likely causes for the severe, accelerated progression of HCV-related cirrhosis [8, 21]. In particular high-dose steroids, immunosuppressive drug combinations, a number of patient co-factors such as diabetes mellitus, baseline demographics, powerful induction treatments, and acute rejection may further promote disease progression [22]. However, the mechanisms underlying accelerated HCV-induced liver damage after OLT are poorly understood. Therefore, the pathogenesis is one of the most important issues in HCV-associated liver fibrosis research after OLT.

Liver fibrosis, developed chronic liver inflammation or injuries, is an excessive deposition of extracellular matrix (ECM) proteins in healing lesions and eventually results in LC. Hepatic stellate cells (HSCs), located in the space of Disse, are the cornerstone of liver fibrosis [23]. HSCs are activated and proliferated to myofibroblast-like cells through the epithelial mesenchymal transition (EMT) and secretion of abundant cytokines and ECM through autocrine and paracrine processes. Besides, activated HSCs also secretes tissue inhibitors of metalloproteinases (TIMPs) degrade ECM. When ECM synthesis outpaces degradation, the resulting superabundant ECM deposition can lead to liver fibrosis [24, 25]. Thus, to estimate whether a factor is protective or detrimental during liver fibrosis, researches could be started by getting a preliminary picture from in vitro co-culture/stimulation experiments with HSCs. Interestingly, under inflammatory circumstances, activated HSCs can also behave as antigen presenting cells and elicit specific cellular responses that modulate the composition of inflammatory infiltrates and the vigor of fibro-genesis [26]. So, investigating the relationship between immune cells and HSCs in HCV-OLT liver fibrosis is a perfect cut-in point to discover indicators for the severity of disease progression.

RETRACTED

Interleukin-22 (IL-22), acting via a heterodimer IL-10R2/IL-22R1 complex, is produced by a variety of hematopoietic cells such as innate lymphoid cells (ILCs), lymphoid tissue-inducers [27], T helper (Th) cells [28] and γδT cells [29]. Meanwhile, IL-22R1 and IL-10R2, receptors of IL-22, are expressed on specific tissues, such as hepatocytes and epithelial cells of gastro-intestine, pancreas, skin, lungs [30–32]. It has been demonstrated that through JAK and STAT molecules, IL-22 appeared to stimulate innate immunity by controlling tissue responses to inflammation, promoting the production of anti-microbial peptides, secreting mucus, releasing chemokine 8–10 and enhancing cell mobility [32–35]. Regarding liver diseases, some studies have shown that IL-22 appeared to be hepatoprotective against CCL_4_, concanavalin A (Con A) and FAS ligand (FasL) injury [36, 37]. On the other hand, compelling evidence also supports that IL-22 plays a potential pathogenic effect in promoting liver tumor cell growth [38, 39]. Recently, several studies have showed that IL-22 is up-regulated in hepatitis B virus (HBV) [39–41] or HCV [42–44] infection and exacerbate chronic liver inflammation and fibrosis in patients and mice [31]. In general, whether this cytokine protects against or aggravates various human diseases is depended on the nature and location of the affected tissues and local cytokine context [34, 45].

However, it is illusive regarding the roles of IL-22 in the progression of chronic liver disease, especially without available information in HCV-OLT. To address these issues, we designed this study to determine the expression, the possible relationship and mechanisms with the disease progression in HCV-OLT patients.

RETRACTED

## Methods

### Ethics Statement

All patients provided the written informed consents for their blood samples, liver biopsy and their information were anonymized. Ethics approval was given by the Medical Ethics Committee of the 302 hospital and the study were in compliance with the Declaration of Helsinki. No conflict of interest during all organ transplantations. No organ trafficking involved (S1 Fig).

### Patients

Fifteen HCV-OLT patients were enrolled into this study in the Department of Liver Transplantation and Research Center of Beijing 302 hospital from June 2010 to September 2014. Data were collected and analyzed on October 2014. All authors listed who were approved by the Medical Ethics Committee of the 302 Hospital, had access to identifying information during or after data collection. All the patients were HCVRNA positive without HCC or other diseases before OLT. No anti-viral therapy before and after transplantation. HCV recurrence was identified HCVRNA positive by quantitative Polymerase Chain Reaction (PCR) (detection limit of 100 IU/mL), anti-HCV Ab positive by Enzyme Linked Immunosorbent Assay (ELISA) and liver histology showing diagnostic pathologic features. Patients were at least six months post-OLT to avoid confounding effect of early post-OLT ischemia-reperfusion injury and surgical complication. Liver biopsies were performed at HCV recurrence and again around two years after recurrence to monitor the progression of diseases. The healthy control group consisted of 15 age- and gender- matched non-HCV post-OLT. Most of the OLT patients underwent induction with methylprednisolone, which was followed by tacrolimus (FK506) and mycophenolate mofetil. Patients between two groups had no significant difference in the median follow-up time and plasma concentration of FK506. The disease control group with similar gender and age distribution to HCV-OLT group was composed of 15 HCV patients, which hadn’t received any antiviral or immunomodulatory therapy. Liver histological tests were conducted in OLT patients for routine follow-up and HCV patients for pathological evaluation. Table 1 lists the clinical and pathological features of the whole patients. In addition to the tissues used for pathological evaluation and embedded for in situ immunohistochemical staining, liver biopsy were immediately frozen and stored in liquid nitrogen for extraction of total RNA and isolation of liver-infiltrating lymphocytes (LILs).

RETRACTED

**Table 1:** Clinical characteristics in different groups.

	OLT	HCV	HCV-OLT
Number (n)	15	15	15
Age (years)	44.7±11.9	41.6±9.4	43.5±13.2
Gender (male/female)	12/3	12/3	12/3
ALT (U/L)	24.6±3.1	63.2±6.5	76.13±5.8
HCV RNA (Log 10 IU/mL)	NA	7.19±0.17	5.6±0.20
HCV Genotype (1b/2a)	NA	8/7	9/6
FK506 (ng/mL)	7.7±1.2	NA	7.4±0.9
Follow-up after OLT (years)	29.7±5.6	NA	28.4±6.5

NA, not applicable; ALT, Alanine aminotransferase; Normal values: ALT, 0–40U/L; Hepatitis C Virus infection (HCV), Hepatitis C Virus recurrence after orthotopic liver transplantation (HCV-OLT), Control cases after orthotopic liver transplantation (OLT)

### Enzyme Linked Immunosorbent Assay (ELISA)

IL-22 (Cat. #D2200, R&D, Minneapolis, MN, US) in serum samples and liver fibrosis markers including Laminin (LN), Hyaluronic Acid (HA) and Collagen type IV (COL IV) (Yuande Biotec, Beijing, China) in the supernatant of *in vitro* cultures were measured by ELISA kits according to the manufacturer’s instructions in triplicate.

### Isolation of LILs

Liver biopsy was homogenized for the isolation of LILs using methods previously described [31, 45]. Briefly, liver tissues were whittled into small pieces after washing with Hank’s solution, and then transferred into Dounceglass tissue grinder and homogenized by gently pestle until no tissue is visible. Dissociated cell suspension was passed through a 70μm Nylon mesh cell strainer (BD Labware) and underlaid onto Ficoll-Hypaque separation solution. LILs were then isolated by density gradient centrifugation.

### Flow Cytometric Analysis

FITC-conjugated Mouse anti-Human CD4 (FITC-CD4) (Cat. 11–0049), PE-conjugated Mouse anti-Human IL-22 (PE-IL-22) (Cat. 12–7229), and Intracellular Fixation/Permeabilization Buffer Set (Cat. 88–8824) were purchased from eBioscience (San Diego, CA, US).

For intracellular IL-22 cells staining, fresh peripheral blood (200ul) and LILs were stimulated with 100 ng/mL phorbol myristate acetate and 1 ug/mL ionomycin (both from Sigma, St. Louis, MO, US) in 800ul RPMI-1640 (Invitrogen, Carlsbad, CA, US) supplemented with 10% heat-inactivated fetal calf serum (FCS) (Gibco, Grand Island, NY, US) for 6h at 37°C in 5% CO_2_ environment. 10 mg/mL Brefeldin A solution (Tocris Cookson, Bristol, UK) was added during the first hour of incubation. The cells were stained surface markers with FITC-CD4, then fixed, permeabilized, and finally stained intracellular markers with PE-IL-22. Using BD fluorescence-activated cell sorting (FACS) CantoTM Ⅱand FlowJo sofrware (TreeStar, Ashland, OR, US) to analyze the cells and the data.

### RNA Isolation and Real-Time PCR (RT-PCR)

Total RNA was extracted using TRIZOL reagent (Invitrogen, Carlsbad, CA, US). Reverse transcription was produced using the SuperScript^TM^ II. Reverse Transcriptase (Invitrogen) and quantitative RT-PCR were conducted with SYBR Green PCR master mix (Applied Biosystems, Foster City, CA, US) following manufacturer’s instructions. Then samples were performed using 7500 RT-PCR System (Applied Biosystems) and assessed in triplicate. Primers for IL-22, α-SMA, TGF-β, TIMP-1 and glyceraldehyde 3-phosphate dehydrogenase (GAPDH) were shown in Table 2.

RETRACTED

**Table 2:** Sequences of oligonucleotides used as primers.

Target gene		Sequence (5’-3’)
IL-22	Forward	TGCATTTGACCAGAGCAAAG
	Reverse	AGTTTGGCTTCCCATCTTCC
α-SMA	Forward	CCGACCGAATGCAGAAGGA
	Reverse	ACAGAGTATTTGCGCTCCGAA
TGF-β	Forward	CCCAGCATCTGCAAAGCTC
	Reverse	GTCAATGTACAGCTGCCGCA
TIMP-1	Forward	CTGTTGTTGCTGTGGCTGATA
	Reverse	CCGTCCACAAGCAATGAGT
GAPDH	Forward	GAAGGTGAAGGTCGGAGT
	Reverse	GAAGATGGTGATGGGATTTC

### Liver Biopsy Measurements

Percutaneous liver biopsies were performed and samples were stained with hematoxylin and eosin, Masson’s trichrome and reticulin staining. The degree of hepatic inflammation and fibrosis was graded using the modified histology activity index (HAI) described by Scheuer [46], which classifies liver fibrosis as absent (F0), restricted to the portal tract (F1), peri-portal or portal-portal septa with intact architecture (F2), bridging fibrosis with architectural distortion but no obvious cirrhosis (F3), and cirrhosis (F4). We defined rapid fibrosis progression (RFP) as liver fibrosis extending beyond the portal tracts (F2-F4) at biopsy 2 (second liver biopsy around two years after HCV recurrence), while slow fibrosis progression (SFP) as fibrosis absent or minimal fibrosis (F0-F1). Mean interval from biopsy 1 to biopsy 2 is 22.7±3.6 months. The minimal acceptable size of liver biopsy was considered 5μm.

### Immunolocalization of IL-22 and α-SMA

Paraffin-embedded, formalin-fixed human liver tissues were incubated with anti-IL-22 (ab18499, abcam, Cambridge, MA, US) or α-SMA antibody (ab7817, abcam) overnight at 4°C followed by heat mediated antigen retrieval with sodium citrate buffer (pH 6.0, 0.1 mol/L) for 20mins and blocking endogenous peroxidase activity with 0.3% H_2_O_2_. Revelation of primary antibody was carried out using horseradish peroxidase (HRP)-conjugated rabbit polyclonal anti-mouse (ab6728, abcam), secondary antibody followed by diamino-benzidine (DAB) and haematoxylin coloration. Double staining was performed with 3-amino-9-ethyl-carbazole (red color) for IL-22 and BCIP/ NBT (indigo color) for CD4. Positively stained cells were counted at high-power field (hpf, ×400) according to described protocols [47].

RETRACTED

### Western Blotting

Liver samples lysis, protein extraction and western blot analysis were performed as previously described [47]. Detection of IL-22 protein was used with mouse anti-Human IL-22 (1 ug/ml, Cat. #AF782, R&D, Minneapolis, MN, US). Protein loading was normalized to GAPDH. The ratio of IL-22 to GAPDH was calculated as the relative quantification.

### Human Hepatic Stellate Cells (HSCs) Stimulation

HSCs, obtained from liver specimens of patients with nonparasitic hepatic cysts who had undergone surgical resections, were isolated, cultured and prepared using methods previously described [48–51]. HSCs cells were directly co-cultured in a U-bottom 96-well plates in triplicate with or without IL-22 at various concentrations (20, 40 ng/mL, PeproTech, London, UK). After incubation for 48h and 72h, cell pellets and supernatants were harvested by centrifugation at 10,000 rpm for 5mins and cell pellets placed in RNALater solution (Ambion), then both cryopreserved at -80°C. Later, the cell pellets were evaluated the expression of α-SMA, TGF-β and TIMP-1 mRNA and supernatant were determined collagen production including LN, HA and COL IV by ELISA.

### HSCs Proliferation and Apoptosis

HSCs were incubated with or without IL-22 at various concentrations (20, 40 ng/mL) for 48h and 72h in the 96-well plates in triplicate. Then cells proliferation was analyzed by testing the concentration of formazan in supernatants using a Cell Counting Kit-8 (CCK-8) commercial kit (Dojindo, Kuma-moto, Japan).

Soluble tumor necrosis factor-related apoptosis-inducing ligand (TRAIL) (20 ng/mL) was added into medium for 6h after incubation of HSCs with or without IL-22 (20 ng/mL) for 48h. Then, cells were resuspended with binding buffer (10mM HEPES/NaOH, pH 7.4, 140mM NaCl, 2.5mM CaCl_2_) and incubated with Annexin V and 7-am-inoactinomycin D (7-AAD) (Biolegend, San Diego, CA, US) for 15mins before analysis using FACS.

### Statistical Analysis

All data were analyzed using SPSS 16.0 statistical software (Version 16.0, SPSS Inc., Chicago, IL, US). Results were expressed as means ± SD. Statistical comparisons between two groups used a Mann-Whitney non-parametric U test, whereas comparisons between the same individual used a Wilcoxon’s matched-pairs t test. The Kruskal-Wallis H nonparametric test was used for multiple comparisons between different groups. The Spearman’s rank correlation test was used to assess the relationship of immune factors and clinical characters. Two-sided P < 0.05 was considered statistically significant.

## Result

### Clinical Characteristics of Different Outcomes of HCV-OLT Patients

Table 3 listed the basic characteristics of HCV-OLT patients pre and postoperatively. Cellular rejection was excluded by histological examination. Mean interval from biopsy 1 to biopsy 2 was 22.7±3.6 months. HCVRNA reappeared within one year and liver biopsy showed absent or minimal fibrosis (F0-F1). However, after two years, eight (53.3%) patients developed severe liver fibrosis; another three patients resulted in liver cirrhosis. The titers of HCVRNA of recurrence were higher than that before OLT (5.60 ±0.20 versus 6.75 ±0.22, p = 0.0006) and significantly lower than that after two years (6.75 ± 0.22 versus 7.39 ±0.16, p = 0.0259). ALT also elevated with progression of HCV-OLT. With respect to genotypes, 9 patients had genotype 1b, and the remaining 6 had genotype 2a. The titers of HCV RNA were similar between HCV-OLT patients with genotype 1b and 2a (p = 0.2874).

RETRACTED

**Table 3:** Virological, serological and clinical features of patients with HCV-OLT.

Number	Pre-OLT		Post-OLT						
	Genotype	HCVRNA	Recurrence (biopsy 1)				After about two year(biopsy 2)		
			time	ALT	S	HCVRNA	S	ALT	HCVRNA
1	1b	5.87	9	58	1	6.49	1	132	7.77
2	1b	5.02	11	97	0	6.24	3	119	6.98
3	2a	5.48	12	82	1	7.18	1	94	7.96
4	1b	6.20	7	76	0	6.98	4	157	7.48
5	2a	4.67	8	71	0	5.13	1	102	7.51
6	2a	4.42	11	64	1	5.32	3	96	6.87
7	1b	6.81	6	85	1	7.35	4	87	8.03
8	1b	6.99	8	89	1	8.00	2	184	6.20
9	1b	6.03	9	56	0	6.87	1	73	7.13
10	2a	5.10	7	51	0	6.98	2	105	6.49
11	1b	4.44	10	115	1	7.51	4	148	7.35
12	2a	5.67	7	93	0	5.86	2	81	7.18
13	1b	5.77	8	48	0	6.86	1	88	8.14
14	1b	5.50	8	92	1	6.47	1	104	7.24
15	2a	5.97	7	65	0	7.96	1	115	8.51

### Serum and Peripheral IL-22 Levels Increased in HCV-OLT Patients

To investigate the expression of IL-22 in different groups, we analyzed the serum IL-22 using ELISA and peripheral IL-22 cells subsets in the total CD4+T cells population using flow cytometry. As shown in Fig 1A, there were significantly higher levels of serum IL-22 in HCV-OLT patients compared to OLT (44.85±3.76 versus 18.12±2.87 pg/ml; p<0.0001) and HCV patients (26.01±3.80 pg/ml; p = 0.0015). No difference between OLT and HCV patients (p = 0.1087). Our previous experiment had determined that CD4 cells were the main cell population dedicated to IL-22 production [31, 52]. Hence, we assessed the characteristics of peripheral IL-22 cells in the total CD4+T cells (Fig 1B) and found that in both HCV-OLT and HCV, the frequencies of IL-22 cells increased significantly compared with OLT (3.41±0.18% versus 1.08±0.12% pg/ml, p<0.0001; 1.62±0.15% versus 1.08±0.12% pg/ml, p = 0.0074) and the IL-22 in HCV-OLT was significantly higher than that in HCV (p<0.0001) patients (Fig 1C). These results suggested that IL-22 cells were markedly accumulated in the liver tissues of HCV-OLT.

RETRACTED

**Fig 1:** Serum levels of IL-22 and frequencies of IL-22 producing cells in the peripheral blood mononuclear cells in different groups. (A) Serum levels of IL-22 (pg/ml) were tested by ELISA in patients with OLT, HCV-OLT and HCV. (B) Representative figures of IL-22 CD4+ staining in different groups. (C) The frequencies of IL-22 (pg/ml) in HCV-OLT patients were significantly higher than that in normal controls OLT and HCV patients. IL-22 also increased significantly in HCV than that in OLT. *P < 0.05, **P < 0.01, ***P < 0.001, **** P < 0.0001, ns p>0.05. Hepatitis C Virus infection (HCV), Hepatitis C Virus recurrence after orthotopic liver transplantation (HCV-OLT), Control post-transplant cases (OLT).

### Intrahepatic IL-22 Increased in HCV-OLT and Correlated with Liver Fibrosis

Meanwhile, we also investigated the roles of IL-22 in the liver. We measured the distribution of IL-22 and the expression of gene and protein in the liver in different groups. IL-22 cells were accumulated mainly in portal areas (Fig 2A) and produced by CD4 cells (Fig 2B). The expressions of IL-22 in the HCV-OLT group were significantly higher than those in the OLT (28.85±2.50 versus 8.52 ±1.11, p<0.0001) and HCV (12.00 ±1.20, p<0.0001) groups (Fig 2C). The expressions of IL-22 mRNA were also significantly up-regulated in the HCV-OLT liver than those in either OLT (3.68 ±0.30 versus 1.87 ±0.18, p<0.0001) or HCV (2.18 ±0.24, p = 0.0007) liver, while no significant difference between OLT and HCV group (P = 0.3118) (Fig 2D). Next, IL-22 proteins were detected by western blotting in the liver. They had the same change tendency with the gene expressions (Fig 2E).

**Fig 2:** Distribution, expression and correlation of IL-22 cells with liver fibrosis in the liver. **(A)** IL-22 positive cells mainly located in portal areas with brownish-yellow color by immunohistochemistry. (B) Immunohistochemistry double staining identities IL-22 cells were produced by CD4 cells in liver tissue. Black arrows indicate double-positive cells. The frequencies of IL-22 cells (C) and the expression of IL-22 mRNA (D) in the liver tissue were significantly higher in HCV-OLT patients, compared to the OLT and HCV patients. (E) Protein in the liver also had the same change by Western-blotting. IL-22 cells are positively correlated with α-SMA (F) and fibrosis staging (G), not with grading score (H) and HCVRNA (I). *P < 0.05, **P < 0.01, ***P < 0.001, **** P < 0.0001, ns p>0.05.

Next, to further detect the relationship between roles of IL-22 and the development of HCV infection, we analyzed the correlations between IL-22 frequencies and liver injury and fibrosis in HCV-OLT and HCV patients. As shown in Fig 2, a significantly positive correlation was found between IL-22 cells frequencies and α-SMA (Fig 2F) (P = 0.0003) or fibrosis staging (Fig 2G) (P = 0.0034). No correlation was found between IL-22 cells frequencies and grading score (P = 0.0631) (Fig 2H) or HCV RNA (P = 0.1345) (Fig 2I).

RETRACTED

### Increase of IL-22 Cells Was Associated with Rapid Fibrosis Progression in HCV-OLT

We also divided HCV-OLT patients into RFP (F2-F4) and SFP (F0-F1) group according to the fibrosis score at biopsy 2. No significance existed in recipient demographics, OLT-related parameters and hepatitis C viral parameters between RFP and SFP (Table 4). Eight (53.3%) patients developed RFP after two years; another three patients were diagnosed liver cirrhosis. As shown in Fig 3, there were no fibrosis in the liver when HCV recurrence (Fig 3A). However, as illustrated by Masson trichrome and reticulin staining (Fig 3B), the progressive fibrosis presented after two years of recurrence. We also found more IL-22 cells were significantly infiltrated in RFP liver tissues (Fig 3D) compared with SRF (Fig 3C), and mainly accumulated in fibrotic septa with the progression of fibrosis. The frequencies of IL-22 were much higher in RFP compared with SFP (39.13±1.90 versus 12.31±1.70, p<0.0001) (Fig 3E). However, there was no significant difference between OLT and SFP groups (12.31 ±1.70 versus 8.52 ±1.11, p = 0.0720).This indicated the possibility that IL-22 cells may had a cell-to-cell contact with activated HSCs. Therefore, we used two colors immunofluorescence to determine IL-22R and α-SMA expression. Results showed IL-22R and α-SMA was co-expressed in the liver tissues of HCV-OLT patients (Fig 3F).

**Fig 3:** Frequencies of IL-22 cells are associated with liver fibrosis in the HCV-OLT patients. (A) Liver histology shows no fibrosis in the livers of patients when HCV recurred. (B) However, after two years, HE, Masson trichrome and reticulin staining illustrate significantly the progressive worsening of liver fibrosis in RFP. Compared with SFP (C), more IL-22 cells were infiltrated in RFP, mainly located in the portal (D). (E) IL-22 frequencies in liver significantly elevated in RFP compared with SFP. No significant difference between OLT and SFP groups. (F) The co-expression of IL-22R and α-SMA was observed in the liver tissues of RFP by immunofluorescence. *P < 0.05, **P < 0.01, ***P < 0.001, **** P < 0.0001, ns p>0.05.

**Table 4:** Comparison of recipient demographics, OLT-related parameters, and hepatitis C viral parameters between RFP and SFP patients.

	RFP (n = 8)	SFP (n = 7)	P Value
Recipient			
Age at OLT	44.8±11.4	42.1±12.7	0.6713
Gender (M/F)	5/1	7/2	0.6593
BMI	24.3±7.6	22.7±9.3	0.7196
OLT-related parameters			
Donor age	47.8±12.1	39.2±11.5	0.1835
Cold ischemia time	7.8±2.4	7.4±2.2	0.7433
Warm ischemia time	38.1±12.7	37.8±13.9	0.9658
Immunosuppression	8.1±0.8	7.3±1.3	0.1687
HCV parameters			
Genotype (1b/2a)	5/3	4/3	0.7513
HCVRNA when recurrence	6.78±0.32	6.71±0.32	0.8782

RETRACTED

### IL-22 Promotes HSCs Proliferation and Activation and Inhibits Apoptosis *In Vitro*

Given IL-22 cells were co-localized with α-SMA+ HSCs in the portal area and positively correlated with liver fibrosis and progression of HCV-OLT, we further investigated the influence of IL-22 in regulating HSCs. We found that Cycloheximide (CHX) could induce Annexin V+ 7-AAD- HSCs apoptosis *in vitro*. Interestingly, the addition of IL-22 (20 ng/mL) significantly inhibited HSCs apoptosis (Fig 4A and 4B) following a 4h incubation with CHX that was markedly reduced in IL-22 pre-treated HSCs (13.61±0.97 versus 6.98±0.70, p<0.0001). Meanwhile, we performed contact co-cultures of primary HSCs in intermediate state respectively with IL-22 at various concentrations for 48h or 72h. Results showed there were significances different in the concentration of formazan which represented proliferation in supernatants between HSCs with or without IL-22 at various concentrations (20, 40 ng/mL) for 48h or 72h (Fig 4C). We also assessed the mRNA expression of HSC-sourced growth factors including α-SMA, TGF-β and TIMP-1 in HSCs, and the concentration of liver fibrosis markers including LN, HA and Collagen IV in the supernatants with or without IL-22 (20, 40 ng/mL) for 48h or 72h. Data indicated that, compared with medium, IL-22 cells dramatically promoted the mRNA expression of α-SMA, TGF-β and TIMP-1 (Fig 5A) and the production of LN, HA and Collagen IV (Fig 5C). Also, the roles were significant stronger with the increasing amount of IL-22 and the prolongation of time. Western blotting also showed the expression of α-SMA and Collagen IV had the same change tendency with their gene expressions.

**Fig 4:** IL-22 *in vitro* inhibits the apoptosis and promotes the proliferation of HSCs. (A) Representative dot plots show the expression of 7-am-inoactinomycin D (7-AAD) and Annexin V in HSCs *in vitro*. Values of Annexin V+ and 7-AAD- represent the percentages of HSCs apoptotic cells. (B) Pooled data indicate that the addition of IL-22 significantly reduces the proportion of apoptotic cells. (C) Pooled data showed the OD value of formazan in HSCs supernatant at various IL-22 concentrations (20, 40 ng/mL) for 48h or 72h. *P < 0.05, **P < 0.01, ***P < 0.001, **** P < 0.0001, ns p>0.05.

**Fig 5:** IL-22 *in vitro* induces the activation of HSCs. (A) The mRNA expression of α-SMA, TGF-β and TIMP-1 in different HSCs groups with or without IL-22 at various concentrations (20, 40 ng/mL) for 48h or 72h. (B) The expression of α-SMA also had the same change with mRNA in different concentrations and time points. (C) The cytokine concentration of laminin, hyaluronic acid and collagen type IV in the supernatants were determined at various concentrations (20, 40 ng/mL). (D) The expression of collagen IV was consistent with gene change.

RETRACTED

## Discussion

IL-22, acting as a potent immune mediator, plays vital roles in many liver diseases [31, 36–44].In current study, we firstly investigated the effect of IL-22 in the patients with HCV recurrence after OLT. The major finding are: (1) Peripheral and intrahepatic expression of IL-22 were significantly elevated in OLT-HCV. (2) IL-22 was associated with the rapid fibrosis progression in HCV-OLT. (3) The up-regulation of IL-22 may further active HSCs to release extracellular matrix, a process likely to be implicated in liver fibrosis.

HCV-related disease remains the leading indication for liver transplantation and HCV recurrence is universal after OLT, especially in the patients who had high viremia before transplant. In general, evasion of the innate immune system is the reason to chronic HCV infection and response of priming of adaptive immune modulate the severity of fibrosis progression. Serum HCVRNA reach levels of pre-OLT titers usually within 4 days after surgery, increase and peak around month 3, and finally attain levels 10- to 100-fold around one year [53]. Liver fibrosis progression during immunosuppressive therapy is extremely accelerated and more rapid than that in non-transplant patients, probably due to a compromised virus-specific Th1 CD4 immune response [54]. In our results, after HCV recurrence, HCVRNA and ALT increased persistently with the progression of HCV-OLT and finally led to the development of liver fibrosis after two years, even three patients resulted in liver cirrhosis.

IL-22, a member of IL10 cytokine family, was discovered in 2000 [55]. Many immune cells, such as CD4 T, CD8 T, NK/NKT, γδT, and macrophages cells, can generate IL-22. Among them, CD4+ T cells are the major sources of IL-22 production in both the liver and peripheral blood [28, 34, 56]. Different from other interleukins, IL-22 is a unique cytokine that regulate the inflammation in IL-22 specific tissues and no any direct roles on immune because its receptors are not expressed on immune cells [32]. The potential role of IL-22 in liver diseases has been intensively studied. In murine models, IL-22 attenuated liver injury [37, 57], prevented hepatic failure [58] and improved hepatic steatosis [57], which suggest a tissue protective function of IL-22 in hepatic disorder. However, the pathophysiological relevance and prognostic potential of serum IL-22 in patients with liver diseases of various etiologies is less clear. Different animal models and patients’ condition lead to different result. In HCV infected patients, many studies reported IL-22 played a pathogenic role in the development of chronic liver diseases [42, 43, 45, 52]. In resolved HCV infection, Matthew et al. [59] found significant production of IL-22 was associated with HCV-antigen-specific induction of CD4+T cell proliferation compared with chronic HCV infection, which suggested IL-22 could be involved in HCV clearance. Although IL-22 doesn’t play direct roles on HCV replication [42], IL-22 productions maybe result in a proinflammatory response to eliminate virus by STAT3 activation and its anti-apoptotic and regeneration promotion effect during HCV recurrence after OLT, especially when HCV virus rapidly increase in immunosuppressive environment. Although several researchers have found IL-22 were up-regulated in HCV-infected patients [42–44, 52], the roles remain obscure in HCV recurrent patients after OLT. Here, we clearly demonstrated that the levels of serum and peripheral blood IL-22 were significantly increased in HCV-OLT patients. In the liver, IL-22-producing cells were accumulated mainly in portal areas and produced by CD4 cells. The expressions of IL-22 in the HCV-OLT were significantly higher than those in the OLT and HCV and IL-22 mRNA was also up-regulated in liver.

RETRACTED

In addition, there are also many different correlations between hepatic IL-22 and liver fibrosis. In mouse experiment, Kong et al. [60] reported IL-22 had anti-fibrotic effects in CCl_4_ mouse models, while Zhao et al. [31] reported pro-fibrotic functions in the HBV Tg mouse model. The difference is due to different models. In Kong’s study, liver fibrosis was induced by acute liver damage resulting from CCL4 administration. IL-22 attenuated acute-damage-driven fibrosis through reducing acute hepatocyte injury. However, in Zhao’s study, progressive liver fibrosis in HBV Tg mouse model they used was driven by T-cells mediated immune response. Overexpression of IL-22 accelerated fibrosis through enhancing chronic inflammation. The roles of anti or pro fibrotic IL-22 depend on its roles of inflammatory protection or damage. In clinic studies, Xiang X et al. reported in chronic hepatitis B virus infected patients, IL-22 and non-ELR-CXC chemokines synergistically provided protection in liver inflammation and fibrosis [41], whereas other clinic studies revealed elevated systemic IL-22 were relevant with the progression of liver fibrosis [31, 52, 61]. In our study, we found IL-22 were significantly positively correlated with α-SMA and fibrosis staging, though not correlated with grading score and HCVRNA. The frequencies of IL-22, which mainly infiltrated in fibrotic septa, were much higher in RFP compared with SFP, whereas there was no significant difference between OLT and SFP. This indicated IL-22 was positively correlated with liver fibrosis and progression in HCV-OLT patients.

RETRACTED

Interestingly, we also found IL-22 immunofluorescence staining was co-localized with α-SMA, a marker for activated HSCs, in the portal area in RFP. Over the past decade, the activation of HSCs into myofibroblasts has always been critical to liver fibrogenesis [23] and recent study revealed that quiescent and activated HSCs could express high levels of IL-22R1 [31, 52, 60, 62, 63]. We therefore designed co-cultures of IL-22 with HSCs to explore exact effects of IL-22 cells responses on HSCs activation and proliferation. In the present study, we have demonstrated that the infiltration of IL-22 cells could exacerbate the progression of liver fibrosis in HCV-OLT patients via the stimulation of HSCs. IL-22 have the potential of promoting HSCs proliferation and activation, and inhibiting apoptosis *in vitro*. Similar to other recent studies [36, 37, 60, 64], we found that IL-22 (20 ng/mL) significantly inhibited HSCs cells apoptosis following a 4h incubation with CHX that was markedly reduced in IL-22 pre-treated HSCs. The reason may be IL-22 activates STAT3, which acts as a key transcriptional factor for cell survival via the induction of the anti-apoptotic genes Bcl-2 and Bcl-xL [60]. Additionally, IL-22 also showed a mitogenic effect on HSCs, which is consistent with other study revealing that IL-22 can promote hepatocyte and liver stem cell proliferation (60, 64). Lastly, our data demonstrated that stimulation of HSCs with IL-22 dramatically resulted in the up-regulation of α-SMA, TGF-β and TIMP-1 mRNA expression and the production of laminin, hyaluronic acid and collagen type IV, thus promoting liver fibrosis progression. Also, the roles were significant stronger with the increasing amount of IL-22 and the prolongation of time. Recent studies [31, 52, 65] on HBV and HCV patients showed increased hepatic IL-22 may induce Th17 migration to aggravate liver fibrosis. So, given the effect of IL-22 between its dual protective and pathogenic roles in human liver diseases, future studies should be focused on the differential roles of IL-22 and IL17 in promoting liver inflammation and fibrosis at various stages of HCV-OLT.

## Conclusion

In conclusion, we suggested that the IL-22 was increased and had significant effects on fibrosis progression in HCV-OLT patients for their influence on liver injury and HSCs function. The characterization of the IL-22 in HCV-OLT by our work paves the way for future researches about fibrosis and immune pathways.

RETRACTED

## Supporting Information

S1 Fig 302 Military Hospital of China Medical Ethics Committee Clinical Study Review Decision. (TIF)
